This article has been retracted.

# Analysis of the Clinical Value of MAGE-A9 Expressions in Cervical Cancer Tissues and PBMC

**DOI:** 10.1155/2022/1417752

**Published:** 2022-06-25

**Authors:** Haipeng He, Jiarui Mi, Yuanyuan Su, Bei Wang, Weiming Wang, Yachai Li, Jin Liu

**Affiliations:** Department of Gynecology, Affiliated Hospital of Hebei University, Baoding, Hebei 071000, China

## Abstract

**Objective:**

The aim of this study is to explore the expressions and clinical significance of melanoma-associated antigen-A9 (MAGE-A9) in cervical cancer tissues and peripheral blood mononuclear cells (PBMC).

**Methods:**

108 patients who were scheduled to undergo cervical conization or extensive hysterectomy between March 2019 and January 2021 due to cervical lesions were selected by convenient sampling. According to postoperative pathological results, the patients were divided into a cervical cancer group (*n* = 64) and cervical intraepithelial neoplasia (CIN) group (*n* = 44). The expression levels of MAGE-A9 mRNA in cervical lesion tissues and PBMC were detected by real-time fluorescence quantitative PCR, and the expression of MAGE-A9 protein in lesion tissues was detected by immunohistochemistry. The correlation between MAGE-A9 mRNA expressions in cancer tissues and PBMC and serum tumor markers in patients with cervical cancer and the relationship between MAGE-A9 protein expression in cancer tissues and clinicopathological characteristics were analyzed, and a receiver operating characteristic curve (ROC curve) was drawn to explore the diagnostic value of MAGE-A9 mRNA expressions in cancer tissues and PBMC on cervical cancer.

**Results:**

The expression levels of MAGE-A9 mRNA in cervical lesion tissues and PBMC in the cervical cancer group were significantly higher than those in the CIN group (*P* < 0.05), and the levels of serum SCC-Ag, CA-125, and CEA were significantly higher than those in the CIN group (*P* < 0.05). The positive rate of the MAGE-A9 protein expression in cervical lesion tissues in the cervical cancer group was significantly higher than that in the CIN group (*P* < 0.05). The expression levels of MAGE-A9 mRNA in cancer tissues and PBMC of patients with cervical cancer were positively correlated with serum SCC-Ag, CA-125, and CEA (*P* < 0.05). The positive rate of the MAGE-A9 protein expression in cervical cancer tissues was related to FIGO stage, tumor diameter, degree of differentiation, lymph node metastasis, and high-risk HPV infection (*P* < 0.05) and was not correlated with age and pathological type (*P* > 0.05). The areas under the ROC curves of MAGE-A9 mRNA in lesion tissue and MAGE-A9 mRNA in PBMC were 0.925 and 0.900 in the diagnosis of cervical cancer (*P* < 0.05).

**Conclusion:**

The expressions of MAGE-A9 in cancer tissues and PBMC of patients with cervical cancer are upregulated, which is related to the levels of serum tumor markers and the progression of disease. MAGE-A9 is expected to become an important marker for the diagnosis of early cervical cancer.

## 1. Introduction

Cervical cancer is a malignant tumor of the reproductive system that occurs in the cervical canal, uterus, and vagina. According to relevant data [1], there are 530,000 new cases of cervical cancer in the world each year, and about 250,000 deaths due to cervical cancer. Life health and quality of life are posed a serious threat and early diagnosis and treatment is the key to improving prognosis. More and more studies have pointed out [2, 3]. The formation and evolution of malignant tumors can be regulated by multiple genes, and exploring the expression of tumor-related antigens and specific antigens has important guiding value for the early diagnosis and treatment of malignant tumors. Melanoma-associated antigen (MAGE) is a group of tumor-specific antigens first discovered in melanoma. It is generally not expressed in normal mature tissues but can be highly expressed in various tumor tissues [4]. MAGE-A9 is one of the members of the MAGE gene subfamily A. It has been found that MAGE-A9 is highly expressed in various malignant tumor tissues such as hepatocellular carcinoma, breast cancer, and colorectal cancer [5, 6]. Reports of it in cervical cancer are rare. This study aims to provide new ideas for early diagnosis and treatment of cervical cancer patients by exploring the expression of MAGE-A9 in cervical cancer tissues and peripheral blood mononuclear cells (PBMC) and its relationship with the clinic-pathological characteristics and prognosis of patients.

## 2. Materials and Methods

### 2.1. General Information

A total of 108 patients undergoing cervical conization or extensive hysterectomy due to cervical lesions who were admitted from March 2019 to January 2021 were selected by convenient sampling. Inclusion criteria were as follows: (1) Married women aged 22–65 years. (2) No radiotherapy, chemotherapy, or immunotherapy before surgery. (3) Postoperative pathologically confirmed cervical cancer or cervical intraepithelial neoplasia (cervical intraepithelial neoplasia), CIN). (4) Voluntarily accepted research, cooperates with inspection, and signs informed consent. Exclusion criteria were as follows: (1) Combined with primary tumors in other parts. (2) Combined with other serious underlying diseases such as immune system diseases and major organ insufficiency. (3) Those who cannot tolerate cervical surgery; history of chemotherapy, or surgery. (5) Mental and cognitive abnormalities. (6) Pregnant or lactating women. The 108 patients were divided into a cervical cancer group (64 cases) and CIN group (44 cases) according to postoperative pathological diagnosis. The age of the cervical cancer group was 36–65 years old, with an average of (52.05 ± 7.80) years old. The International Federation of Obstetrics and Gynecology (FIGO) staged [7] 43 cases of stage I, 21 cases of stage IIA; the CIN group aged 25 to 50 years, mean (33.91 ± 6.31) years old stages 15 cases of CIN stage II, 29 cases of stage III. This study complies with the ethical principles of medical research in the Declaration of Helsinki. There are no statistical differences in clinical baseline data between patients in the cervical cancer group and the cervical intraepithelial neoplasia (CIN) group.

### 2.2. Methods

#### 2.2.1. MAGE-A9 mRNA Expression in Cervical Lesions and PBMC

The fresh postoperative cervical lesion tissue samples were collected with sterile EP tubes, placed in a liquid nitrogen tank, and stored at −80°C for future use; we take 0.1 g tissue specimens from EP tubes, grind them into powder repeatedly under liquid nitrogen, and extract total RNA from PBMCs by the TriZOL method. Reverse transcription kit instructions and kits were purchased from Beijing Soleibao Technology. The target gene was amplified using a Roche LightCycler 96 real-time PCR instrument. The primer sequences were synthesized by Shanghai Sangon Bioengineering Co., Ltd. The upstream and downstream primer sequences of MAGE-A9 gene were 5′-CACTGTATGTCATCTCTG-3′, 5′-ACTACTGTCATTCATTAA-CT-3′. Using U6 as the internal reference gene, the upstream and downstream primer sequences are 5′-CTCGCT-TCGGCAGCACA-3′, 5′-AACGCTTCACGAATTTGCGT-3′. PCR reaction conditions: preheating at 95°C for 3 min, denaturation at 95°C for 30 s, annealing at 60°C for 30 s, extension at 70°C for 30 s, a total of 40 cycles, and a final extension at 72°C for 10 min. After the reaction product was electrophoresed on a 2% agarose gel, the optical density of each band was determined by the Gel-Doc XR automatic gel imaging system of Bio-Rad Company. The relative expression of the target gene was calculated using the 2^−△△ct^ method. 5 mL of fasting cubital venous blood was collected by an EDTA anticoagulation tube and centrifuged at 3000 r/min and 8 cm radius for 15 min to separate serum for use; a Percoll cell separation medium (Beijing Soleibao Technology Co., Ltd.) was used to separate PBMCs by density gradient centrifugation. The total RNA of PBMCs was extracted by the TriZOL method. -A9 mRNA detection was consistent.

#### 2.2.2. MAGE-A9 Protein Expression in Cervical Lesions

The expression of MAGE-A9 protein in cervical lesions was detected by the immune-histochemical SP method. The lesion tissue was made into a paraffin block for use, and the paraffin was taken, including 4 *μ*m serial sections, baked in an incubator at 60°C for 20 min, and then graded I (soaked for 10 min), grade II (soaked for 10 min), and grade III in xylene. (soaking for 5 min) dewaxing treatment; placed in gradient alcohol (soaked in anhydrous alcohol twice for 5 min, 95%, 90%, 80%, 70%, 50% alcohol for 5 min each) after dehydration treatment, soaked in flowing distilled water for 10 min, and then immersed in PBS solution. It is rinsed 2 times for 3 min each; placed in 3% H_2_O_2_ solution, incubated at room temperature for 10 min, and then rinsed with PBS twice, 3 min each. Using EDTA repair solution, it was repaired in a microwave oven on high heat for 15 min, cooled to room temperature naturally, and then rinsed with PBS solution 3 times for 5 min each; 1 drop of serum working solution was added dropwise to each section and placed at room temperature for 10 min. Each drop has a primary antibody working solution (mouse anti-human MAGE-A9 primary antibody from Novus, USA) and PBS instead of primary antibody was used as control and incubate it at 4°C; Secondary antibody anti-mouse antibody was incubated at room temperature for 15 min and rinsed 3 times with PBS for 5 min . Each section was dripped with a horseradish peroxidase marker, incubated at room temperature for 10 min, and washed with PBS three times, each for 5 min. Each section was dripped with freshly prepared DAB solution for color development, counterstained with hematoxylin, and then dehydrated with gradient alcohol in sequence. Xylene is then cleared 3 times for 10 min each. Slides are sealed with a neutral gum and read under a light microscope. 5 fields of view (≥100 cells) are randomly selected under a 400x microscope and counted by 2 experts with extensive diagnostic experience. Pathologists made independent judgments after double-blind reading of the films and reached a consensus through consultation when the results were inconsistent. MAGE-A9 protein is mainly stained in the cytoplasm. ①Staining intensity: no staining, light yellow, brownish yellow, and yellowish brown, respectively, scored 0, 1, 2, and 3 points. ②Proportion of positive cells: the proportion of positive cells is less than or equal to 5%, 6%∼25%, 26%∼50%, 51%∼75%, and >75% were scored as 0, 1, 2, 3, and 4 points, respectively; the product of ① × ② product of 0∼1 was considered negative (−), 2∼4 points are weakly positive (+), 6 points or 8 points are positive (++), and 9 points or 12 points are strongly positive (+++), and the product of ① × ② in this study is ≥ 2 points were regarded as positive expression.

#### 2.2.3. Serum Tumor Markers

3 ml of fasting cubital venous blood samples was collected from patients in the morning before surgery, centrifuged at 3000 r/min and a radius of 8 cm for 15 min, and the supernatant was collected for use. The expression of serum squamous cell carcinoma-associated antigen (SCC-Ag), carbohydrate antigen 125 (CA-125), and carcino embryonic antigen (CEA) was detected by the Roche tumor marker kit level; the kit was purchased from Shanghai Yaji Biotechnology Co., Ltd., and the detection steps were operated according to the kit instructions. The normal reference value range of SCC-Ag is 0∼1.5 ng/mL, CA-125 is 0∼35 U/mL, and CEA is 0∼5 ng/m.

### 2.3. Statistical Analysis

The date analysis was processed by SPSS 17.0 software, normal measurement data are listed as ($\bar{x}\pm s$), and independent sample *t*-test was performed; count data were expressed as (*n* (%)), and *χ*2 test was used, and grade data were subjected to two independent samples *t*-test; the Pearson correlation analysis was used for analysis; a receiver operator characteristic curve (ROC curve) was drawn to explore the diagnostic value; *P* < 0.05 was regarded as a significance threshold.

## 3. Result

### 3.1. Comparison of MAGE-A9 mRNA and Serum Tumor Marker Expressions between the Two Groups

The expression levels of MAGE-A9 mRNA in cervical lesion tissues and PBMC in the cervical cancer group were significantly higher than those in the CIN group (*P* < 0.05), and the levels of serum SCC-Ag, CA-125, and CEA were significantly higher than those in the CIN group (*P* < 0.05) as shown in Table 1.

### 3.2. Comparison of the MAGE-A9 Protein Expression between the Two Groups

There was a statistically significant difference in the expression of MAGE-A9 protein in cervical lesions between the two groups and the positive rate of MAGE-A9 protein in the cervical cancer group was significantly higher than that in the CIN group (*P* < 0.05) as shown in Table 2.

### 3.3. Correlation between the MAGE-A9 mRNA Expression and Serum Tumor Markers in Cervical Cancer

The results of the Pearson correlation analysis showed that MAGE-A9 mRNA expression levels in cancer tissues and PBMCs of patients with cervical cancer were positively correlated with serum SCC-Ag, CA-125, and CEA (*P* < 0.05) as shown in Table 3.

### 3.4. Relationship between the MAGE-A9 Protein Expression and Clinic-Pathological Features in Cervical Cancer Tissues

The positive rate of the MAGE-A9 protein expression in cervical cancer tissues was significantly higher in FIGO stage IIA than in stage I, tumor diameter ≥ 3 cm was significantly higher than that of <3 cm, poorly differentiated was significantly higher than well-differentiated, with lymph nodes. The patients with metastases were significantly higher than those without lymph node metastasis, and those with high-risk HPV infection were significantly higher than those without high-risk HPV infection, with statistical significance (*P* < 0.05). However, there was no significant difference in the positive expression of MAGE-A9 protein among different ages and pathological types (*P* > 0.05) as shown in Table 4.

### 3.5. The Value of the MAGE-A9 mRNA Expression in Cervical Cancer Tissues and PBMC in the Diagnosis of Cervical Cancer

Taking the diagnosis of cervical cancer as the state variable, and the expression levels of MAGE-A9 mRNA in the lesion tissue and MAGE-A9 mRNA in PBMC as the test variable, the ROC curve was drawn. The areas under the ROC curve were 0.925 and 0.900 (*P* < 0.05), respectively, and the optimal cutoff values were 0.900 and 1.055, respectively, as shown in Figure 1 and Table 5.

## 4. Discussion

Although the current HPV vaccine promotion, cervical cancer screening, and development of diagnosis and treatment technologies have brought the morbidity and mortality of cervical cancer under a certain control, it is still the malignant tumor with the highest morbidity and mortality in the female reproductive system [8]. At present, the etiology and pathogenesis of cervical cancer have not been fully elucidated. It is often considered the result of multifactor, multistep, and long-term effects. Infections such as HPV and cytomegalovirus are the main microbial pathogenic factors. Family history, unclean sexual life, marriage and birth factors, malnutrition, smoking, etc., are common high-risk factors; in addition, genetic mutations, hormone changes, and other factors are also related to its occurrence and development [9]. Early diagnosis and treatment is key to improving cervical cancer prognosis, but in practice, most patients are already in advanced stages when they are discovered due to the lack of specific symptoms of early cervical cancer. Exploring sensitive biological markers related to the occurrence and development of cervical cancer can provide early clinical diagnosis and treatment. Therefore, related research has attracted much attention [10].

MAGE is a member of the cancer/testis antigen family. Since it was first isolated and cloned from melanoma in 1991, at least 13 subfamilies and 83 closely related gene members of the MAGE family have been found [11]. In general, MAGE is mainly manifested in the testicles and placenta, but it is widely and highly expressed in a variety of malignant tumors and has a certain correlation with tumorigenesis, development, drug resistance, and prognosis [12]. MAGE-A9 is one of the most studied members of the current MAGE family. It is located on the Xq28 chromosome. The full-length cDNA is 945 bp. The molecular weight of the encoded protein product is about 35 ku. Peptides are involved in tumor T cell immune responses, and MAGE-A family members have high homology, so MAGE-A9 is expected to be a potential target for tumor biological immunotherapy [13]. Studies have pointed out that the expression of MAGE-A9 protein in laryngeal squamous cell carcinoma is significantly increased, and it is related to the clinical stage and lymphatic metastasis of patients [14]. It is considered to be a prognostic indicator of laryngeal squamous cell carcinoma. It has been reported in the literature [15] that MAGE-A9 protein is highly expressed in human non-small-cell lung cancer cell lines, and downregulation of the MAGE-A9 expression by RNAi technology can reduce cell migration and invasion, so MAGE-A9 is closely related to non-small-cell lung cancer. It is related to the development process of lung cancer migration and invasion. At present, there are not many reports on MAGE-A9 in the female reproductive system malignant tumors. Some researchers pointed out that the expression of MAGE-A9 protein in ovarian cancer tissues was significantly upregulated, which was significantly correlated with FIGO stage, histological grade, and tumor metastasis of ovarian cancer [16]. The MAGE-A9 expression is an independent factor affecting the prognosis of ovarian cancer patients. In addition, the overexpression of MAGE-A9 can enhance the malignant biological ability of ovarian cancer cell lines, and interference with its expression can inhibit the proliferation, migration, and invasion of ovarian cancer cells and improve the sensitivity of cisplatin chemotherapy. Therefore, the MAGE-A9 expression shows an application value in ovarian cancer prognosis prediction and targeted therapy. In this study, real-time fluorescence quantitative PCR was used to detect the expression of MAGE-A9 mRNA in cervical lesion tissues and PBMC of cervical cancer and CIN patients. The immunohistochemical SP method was used to detect the expression of MAGE-A9 protein in cervical lesions. It was found that the positive rate of the MAGE-A9 protein expression in the cervical cancer group was significantly higher than that in the CIN group. Therefore, it is speculated that the MAGE-A9 expression is upregulated in cervical cancer patients. Further analysis found that the positive rate of MAGE-A9 protein expression in cervical cancer tissues was related to FIGO stage, tumor diameter, degrees of differentiation, lymph node metastasis, and high-risk HPV infection. Therefore, it is speculated that MAGE-A9 is involved in the occurrence, invasion, and metastasis of cervical cancer. This is similar to some reports [17]. Studies have pointed out that MAGE-A9 may participate in the progression of malignant tumors by inhibiting the transcriptional activity of the tumor suppressor gene p53, interfering with its biological functions such as inhibiting malignant proliferation and promoting apoptosis [18].

However, the mechanism by which MAGE-A9 participates in the occurrence and development of cervical cancer is still unclear, and the relevant mechanism remains to be explored by more basic research. CEA is a broad-spectrum tumor marker that is useful for predicting recurrence and survival rates in many carcinomas, such as colon or gastric cancer. Moreover, when combined with carbohydrate antigen 19–9 (CA19-9), the level of CEA is closely correlated with the survival of patients with non-small-cell lung cancer. CA125 is considered a potential marker for ovarian cancer, and the combined detection of CA125 and human epididymis protein 4 (HE4) is effective for screening non-small-cell lung cancer. These markers are also closely related to lung cancer, and most of the studies focused on the predictive value of these markers for prognosis and survival rate in lung cancer. These results suggest that these markers are important for prognosis and survival assessment. In addition, this study also found that the areas under the ROC curve of MAGE-A9 mRNA in lesion tissues and MAGE-A9 mRNA in PBMC for the diagnosis of cervical cancer were 0.925 and 0.900, respectively, and were positively correlated with serum SCC-Ag, CA-125, and CEA of patients, suggesting that the detection of MAGE-A9 mRNA may provide a reference for the early diagnosis and treatment of cervical cancer, which is worthy of further exploration. The disadvantage of this study is that due to the limitation of follow-up time, the relationship between the MAGE-A9 expression and prognosis of cervical cancer patients has not been further explored.

In conclusion, the expression of MAGE-A9 in cancer tissues and PBMC of patients with cervical cancer was significantly increased, which was correlated with the level of serum tumor markers in patients and was related to tumor stage and metastasis. The study provides reference for early diagnosis of cervical cancer.

## Figures and Tables

**Figure 1:** The ROC curve of MAGE-A9 mRNA in cervical cancer tissues and PBMC in the diagnosis of cervical cancer.

**Table 1:** Comparison of the MAGE-A9 mRNA expression and serum tumor markers between the two groups ($\bar{x}\pm s$).

Group	*n*	MAGE-A9 mRNA		Tumor markers in serum		
		Lesion tissue	PBMC	SCC-Ag (ng/mL)	CA-125 (U/mL)	CEA (ng/mL)
Cervical cancer group	64	1.321 ± 0.482	1.726 ± 0.513	3.96 ± 1.66	49.20 ± 15.01	13.71 ± 5.19
CIN group	44	0.601 ± 0.188	0.942 ± 0.321	0.70 ± 0.35	25.57 ± 8.16	3.09 ± 1.33
*T*		9.426	8.990	12.812	9.515	13.272
*P*		<0.001	<0.001	<0.001	<0.001	<0.001

*P* < 0.001 was regarded as a significance threshold.

**Table 2:** Comparison of the MAGE-A9 protein expression between the two groups (*n* (%)).

Group	*n*	MAGE-A9				
		−	+	++	+++	Positive rate
Cervical cancer group	64	23 (35.94)	12 (18.75)	19 (29.69)	10 (15.62)	41 (64.06)
CIN group	44	34 (77.27)	7 (15.91)	3 (6.82)	0 (0.00)	10 (22.73)
*Z/χ* ^*2*^	4.64					17.875
*P*	<0.001					<0.001

*P* < 0.001 was regarded as a significance threshold.

**Table 3:** Correlation between the MAGE-A9 mRNA expression and serum tumor markers in cervical cancer.

Index	SCC-Ag		CA-125		CEA	
	*r* value	*P* value	*r* value	*P* value	*r* value	*P* value
MAGE-A9 mRNA in cancer tissue	0.644	<0.001	0.320	0.010	0.294	0.018
MAGE-A9 mRNA in PBMC	0.477	<0.001	0.386	0.002	0.270	0.031

**Table 4:** Relationship between the MAGE-A9 protein expression and clinic-pathological characteristics in cervical cancer tissues.

Indexes		Number of cases	Number of the positive cases	Positive rate (%)	*χ* ^*2*^	*P*
Year (old)	≤50	27	16	59.26	0.468	0.494
	>50	37	25	67.57		

FIGO phase	Phase I	43	23	53.49	6.365	0.012
	Phase IIA	21	18	85.71		

Pathological type of tumor	Squamous cell carcinoma	54	37	68.52	2.981	0.084
	Adenocarcinoma	10	4	40.00		

Diameter of tumor (cm)	<3	51	29	56.86	5.653	0.017
	≥3	13	12	92.31		

Degree of tumor differentiation	Highly differentiated	19	8	42.11	8.294	0.016
	Moderate differentiation	28	18	64.29		
	Poorly differentiated	17	15	88.24		

Lymph node metastasis	Yes	18	16	88.89	6.705	0.010
	No	46	25	54.35		

High-risk HPV infection	Yes	52	37	71.15	6.058	0.014
	No	12	4	33.33		

Human papillomavirus (HPV).

**Table 5:** The diagnostic value of MAGE-A9 mRNA in cervical cancer tissues and PBMC for cervical cancer.

Indexes	Area	Standard error	*P*	95% CI		Cutoff value	Sensitivity	Specificity
				Lower bound	Upper limit			
MAGE-A9 mRNA in lesion tissue	0.925	0.025	<0.001	0.875	0.974	0.900	0.797	0.955
MAGE-A9 mRNA in PBMC	0.900	0.029	<0.001	0.843	0.958	1.055	0.938	0.750

## Data Availability

The raw data supporting the conclusion of this article will be available by the authors without undue reservation.
